# Effects of Stress Psychological Intervention on the Cardiopulmonary Function, Negative Emotion, Self-Efficacy, and Quality of Life in Patients with Acute Respiratory Failure

This article has been retracted.

**DOI:** 10.1155/2021/9359102

**Published:** 2021-09-13

**Authors:** Na Zhu, Fang Gu, Yiqian Hu, Wen Bian

**Affiliations:** ^1^Emergency Intensive Care Unit, Affiliated Hospital of Jiangnan University, Wuxi, Jiangsu 214000, China; ^2^Emergency General Ward, Affiliated Hospital of Jiangnan University, Wuxi, Jiangsu 214000, China; ^3^Emergency Department, Affiliated Hospital of Jiangnan University, Wuxi, Jiangsu 214000, China

## Abstract

**Objective:**

To investigate the changes in cardiopulmonary function, negative emotion, self-efficacy, and quality of life in patients with acute respiratory failure (ARF) after stress psychological intervention.

**Methods:**

A prospective study was conducted on 104 patients with ARF admitted to our hospital from March 2019 to March 2021. According to the random number method, the patients were divided into a control group (*n* = 52) and an experimental group (*n* = 52). Routine intervention was implemented in the control group, and stress psychological intervention was implemented in the experimental group on the basis of the control group. The cardiopulmonary function, negative emotion, self-efficacy, and quality of life in the two groups were compared.

**Results:**

The left ventricular ejection fractions and fraction shortening in the experimental group were higher than those in the control group, as well as the left ventricular mass index was lower than that in the control group (*P* < 0.05). The first forced expiratory volume (FEV_1_), forced vital capacity (FVC), and FEV_1_/FVC in the experimental group were higher than those in the control group (*P* < 0.05). The Self-Rating Anxiety Scale scores and Self-Rating Depression Scale scores in the experimental group were lower than those in the control group (*P* < 0.05). The General Self-Efficacy Scale scores of the experimental group were higher than those of the control group (*P* < 0.05). The Concise Health Measurement Scale scores of the experimental group were higher than those of the control group (*P* < 0.05).

**Conclusion:**

Stress psychological intervention in patients with ARF can improve cardiopulmonary function, reduce negative emotions, improve self-efficacy, and improve quality of life.

## 1. Introduction

Acute respiratory failure (ARF) is a disease of the body's lung ventilation and/or ventilation dysfunction in a short period of time, which can be caused by obstructive pulmonary emphysema, asthma, sleep apnea syndrome, and other various reasons [1]. ARF often leads to insufficient oxygen supply and carbon dioxide retention in the body of patients, making the body unable to carry out effective gas exchange, and is prone to hypoxemia or hypercapnia and even causes ischemia and hypoxia of other organs, resulting in multiple organ failure [2]. The main clinical manifestations of ARF patients are dyspnea, increased blood pressure, skin congestion, increased sweat, increased heart rate, and other manifestations and may be accompanied by symptoms such as cyanosis, convulsions, and coma, which can cause serious damage to the patients' organ function and bring great inconvenience to the life of the patients [3, 4]. During the period of treatment and rescue, patients with ARF are often prone to produce relatively strong psychological stress response due to the acute onset of the disease, the pain of the treatment, the doubt about the treatment effect, the uncertainty about the outcome of their own disease, the fear of death, the unfamiliar environment, and other stressor [5]. Stress psychological response refers to an unhealthy state of the body caused by the imbalance of objective requirements and coping ability under a certain stimulus [6]. When patients with ARF have a stress psychological response, they will not only produce various psychological problems such as anxiety and depression, which will reduce the patients' sense of self-efficacy, but also reduce the patients' degree of cooperation in treatment, so that they will resist treatment and nursing activities, which will affect the rescue and recovery of the disease and then reduce the patients' living standards [7]. With the rapid onset and rapid changes of ARF, it has great difficulties and problems in clinical nursing. With the improvement of the social level, people's requirements for medical services are increasing. Therefore, finding more scientific and reasonable intervention measures is crucial to the recovery of patients, which can help patients with ARF to eliminate or adapt to stressors as soon as possible.

In recent years, stress psychological intervention has been gradually applied to a variety of clinical diseases and has been favored by people. Stress psychological intervention takes the patients' own perspective as the entry point. Through the implementation of psychological interventions such as psychological diagnosis, understanding, communication, and re-education, it can stabilize the patients' emotions, overcome the psychological crisis, reduce the stress response, and further ensure the smooth progress of treatment [8]. The research by Antoni and Dhabhar [9] showed that chronic stress, painful state, and other social and psychological stress factors will affect the immune variables in cancer, and the implementation of psychological intervention and stress management intervention for cancer patients can improve the clinical disease status of patients. Barreau [10] reported that patients with renal failure often have multiple psychological effects during hemodialysis and may experience acute psychological crises; therefore, it is necessary to carry out effective psychological interventions for hemodialysis patients in clinical practice.

At present, stress psychological intervention plays a dominant role in holistic care, but the relevant research on the application of this intervention mode to patients with ARF is relatively rare. Therefore, this study aims to analyze the effect of stress psychological intervention on the cardiopulmonary function, negative emotion, self-efficacy, and quality of life of patients with ARF in order to provide a basic theoretical basis for the selection of clinical nursing programs.

## 2. Materials and Methods

### 2.1. Research Object

A prospective study was conducted on 104 patients with ARF admitted to our hospital from March 2019 to March 2021. Patients were grouped according to the random number method. Patients who met the criteria were numbered according to the date of admission, starting with any number in a random number table, each patient was assigned a random number in the same direction, and the odd numbers were entered into the experimental group and even numbers into the control group. Finally, according to this method, the patients were divided into a control group (*n* = 52) and an experimental group (*n* = 52).

#### 2.1.1. Diagnostic Criteria

① There were causes of pulmonary ventilation and/or ventilation dysfunction. ② There were clinical manifestations related to hypoxia and carbon dioxide retention, such as dyspnea, cyanosis, neuropsychiatric symptoms, cardiovascular system manifestations, and blood circulation symptoms. ③ Under the conditions of sea level, resting state, and breathing air, arterial blood oxygen partial pressure (PaO_2_) <60 mmHg with or without carbon dioxide partial pressure (PaCO_2_) >50 mmHg and the factors causing hypoxia such as intracardiac anatomic shunt and primary cardiac output reduction were excluded. ④ The diagnosis was confirmed by ordinary chest X-ray, chest CT, and other imaging examinations.

#### 2.1.2. Inclusion Criteria

It met the diagnostic criteria of ARF [11]; the course of the disease was less than 12 h; the consciousness was clear, and the basic understanding or expression ability; the condition of oneself was known; and the clinical data were completed.

#### 2.1.3. Exclusion Criteria

Accompanied by other serious diseases, mentally ill, abnormal hearing, poor compliance, and withdrawing midway.

### 2.2. Research Methods

#### 2.2.1. Control Group

Routine intervention was implemented after admission. Quickly found out the cause of the patient's disease and evaluated the patient's condition. The principle of first aid was to immediately open the airway, gave the medicine as prescribed by the doctor, and closely observed the changes in the condition after the first aid to keep the airway unobstructed and promote respiratory recovery. The intervention lasted for 2 weeks.

#### 2.2.2. Experimental Group

On the basis of the control group, stress psychological intervention was carried out. A stress psychological intervention team, which was composed of head nurses, specialist nurses, and psychological counselors who had undergone professional learning, was established. Division of membership: the head nurse and the specialist nurse jointly formulated the inclusion and exclusion criteria and psychological intervention plan for patients; the specialist nurse was responsible for the collection, analysis, and processing of patients' data; the psychological counselors were responsible for the assessment of patients' psychological status and formulated the detailed psychological intervention content of stress. Before the intervention, the team members all received professional guidance, mastered the specific content of the stress psychological intervention, the method of filling in the questionnaire, and precautions, and formulated a specific intervention plan according to the patient's situation. The intervention lasted for 2 weeks. The specific method was as follows. ① Diagnosis: Medical staff should actively communicate with patients as much as possible, enhance their sense of trust and cooperation, and establish a good doctor-patient relationship with patients with ARF. They asked the subjective feelings of patients, understood the actual situation of patients, expressed understanding of the current situation of patients, looked for the essential needs of the patients with ARF, confirmed the psychological and behavioral problems of patients, and focused on the analysis and discussion of the reasons for the unreasonable problems. ② Understanding: Used simple and easy-to-understand language to introduce disease knowledge to patients in detail, and used a meticulous and gentle attitude to explain the occurrence of APF, treatment process, prognosis, matters needing attention, and other content, so as to encourage patients to master the whole process of treatment and nursing. In view of different psychological states of patients, in-depth conversation was conducted to help patients realize the occurrence of their own bad emotions and abnormal behavior symptoms, guided them to understand the importance of correct cognition and behavior, and make them realize the wrong cognition and thinking. ③ Communication: Communicated with the patient according to the patient's condition and psychological changes, encouraged the patient to express their inner thoughts, and tried their best to meet the reasonable requirements of the patient. By means of practical verification, the patients' wrong ideas were changed, the patients were guided to master the correct treatment thoughts, and the corrected outlook on the life and world could be established, so as to alleviate the psychological pressure of the patients. Using body language to comfort patients helped the patients get psychological support and comfort, so as the degree of treatment coordination was improved. Regular communication training was conducted for the patients' families, explained the importance of family support to the patients' families members, and urged the family members to pay more attention to the patients' disease and mental state, communicate with the patients more, and help the patients to have a positive concept. ④ Re-education: Explained in detail the psychological impact of the disease on the patients' progress, strengthened the cultivation of patients' rational concepts, and further eliminated irrational concepts. In view of the patient's existing psychological problems, the medical staff re-adjusted the patient's psychology, instructed the patient to establish a healthy attitude, and caused the patient to accept the occurrence of the disease. Helped patients recall happy things in life and encouraged patients to participate in outdoor activities or listen to more relaxing music, so that patients kept their body relaxed and happy.

### 2.3. Research Tools

Both groups of patients were evaluated for treatment effect after 2 weeks of intervention. A uniformly trained researcher gave guidance to the research objects, explained the purpose and precautions of the research, and conducted the survey by filling in a questionnaire. The effective recovery rate of the questionnaire was 100%.

#### 2.3.1. Clinical Data

The clinical data such as age, gender, type (type was performed by arterial blood gas analysis), cause of disease, and level of education were recorded.

#### 2.3.2. Cardiac Function

The Philips EPIQ5 full-digital thinking color Doppler ultrasound system was used to detect left ventricular ejection fractions (LVEF), left ventricular fraction shortening (FS), and left ventricular mass index (LVMI) of the two groups.

#### 2.3.3. Lung Function

The spirometer was used to detect the first forced expiratory volume (FEV_1_), forced vital capacity (FVC), and FEV_1_/FVC (the ratio of the first forced expiratory volume to the forced vital capacity) of the two groups.

#### 2.3.4. Negative Emotions

Self-Rating Anxiety Scale (SAS) [12] and Self-Rating Depression Scale (SDS) [13]: Both had 20 items and adopted a 4-level scoring method. An SAS score of <50 points indicates no anxiety, 50–59 points indicates mild anxiety, 60–69 points indicates moderate anxiety, and >69 points indicates severe anxiety. An SDS score of <53 points indicates no depression, 53–62 points indicates mild depression, 63–72 points indicates moderate depression, and >73 points indicates major depression. A higher score indicates more negative emotions. Cronbach's *α* coefficient of SAS was 0.802. Cronbach's *α* coefficient of SDS was 0.807.

#### 2.3.5. Self-Efficacy

General Self-Efficacy Scale (GSES) [14]: It had a total of 10 items and adopted a 4-level scoring method. The total score was 10–40 points, with 10–20 points for low efficiency, 21–30 points for medium efficiency, and 31–40 points for high efficiency. A higher score indicates better self-efficacy. Cronbach's *α* coefficient of GSES was 0.869.

#### 2.3.6. Quality of Life

Concise Health Measurement Scale (SF-36) [15]: It had a total of 36 items, including 8 dimensions such as physical function, physical function, physical pain, general health, energy, social function, emotional function, and mental health, and an additional health change, and the score of each dimension was 0–100 points. The average score of each dimension was calculated. A higher score indicates a higher quality of life. Cronbach's *α* coefficient of SF-36 was 0.865.

### 2.4. Statistical Methods

SPSS22.0 software was used for analysis, measurement data were expressed as mean ± standard deviation, and the *t*-test was used for comparison. Count data were expressed as %, and the *χ*^2^ test was used for comparison. *P* < 0.05 was statistically significant.

## 3. Results

### 3.1. Comparison of Clinical Data between the Two Groups

There were no significant differences in age, gender, type, cause of disease, and level of education between the two groups (*P* < 0.05). See Table 1.

### 3.2. Comparison of Cardiac Function between the Two Groups

After intervention, the LVEF and FS of the two groups were higher than those before intervention, and the LVMI of the two groups were lower than that before intervention. The LVEF and FS in the experimental group were higher than those in the control group, and the LVMI was lower than that in the control group (*P* < 0.05). See Figure 1.

### 3.3. Comparison of Lung Function between the Two Groups

After intervention, the FEV_1_, FVC, and FEV_1_/FVC of the two groups were higher than those before intervention, and the FEV_1_, FVC, and FEV_1_/FVC in the experimental group were higher than those in the control group (*P* < 0.05). See Figure 2.

### 3.4. Comparison of Negative Emotions between the Two Groups

After intervention, the SAS scores and SDS scores of the two groups were lower than those before intervention, and the SAS scores and SDS scores in the experimental group were lower than those in the control group (*P* < 0.05). See Figure 3.

### 3.5. Comparison of Self-Efficacy between the Two Groups

After intervention, the GSES scores of the experimental group was higher than those before intervention, and the GSES scores of the experimental group was higher than those of the control group (*P* < 0.05). See Figure 4.

### 3.6. Comparison of Quality of Life between the Two Groups

After intervention, the SF-36 scores of the two groups were higher than those before intervention, and the SF-36 score in the experimental group were higher than those in the control group (*P* < 0.05). See Figure 5.

## 4. Discussion

ARF is often caused by pulmonary and bronchial diseases and ventilatory dysfunction. It mostly occurs in middle-aged and elderly people and poses a serious threat to the life safety of patients [16]. Affected by a variety of factors, patients with ARF are prone to a series of negative emotions such as anxiety, depression, and tension and produce stress psychological reactions, thereby reducing the patients' treatment compliance. If the effective intervention of ARF patients cannot be carried out in time, it may directly affect the implementation and effect of clinical treatment, which is not conducive to disease recovery [17]. Therefore, the application of effective intervention programs to improve the psychological status of patients has a key role.

At present, the routine clinical intervention methods play a certain role in the nursing of ARF patients, but their intervention content is relatively simple and it is easy to ignore the actual situation and psychological conditions of the patients, thus lacking pertinence and initiative and hence failing to achieve the desired nursing effect. Stress psychology is mainly the process of physiological and psychological changes when the body responds to stressors [18]. Jentsch and Wolf [19] found that the nervous system promotes arginine and adrenal cortex hormones to produce stress-regulating effects by regulating the norepinephrine sympathetic system. Therefore, when people have bad psychological stress, the body's neuroendocrine function will change, and the psychological intervention of stress on people can effectively improve the neuroendocrine function and reduce the psychological stress response. Witek's team [20] believed that once people's stress occurs, it will affect the production of helper *T* cells and the immune function will change accordingly. The implementation of mindfulness decompression therapy for women with breast cancer can not only improve the psychological problems but also optimize immune function that supports cancer control. Physicians in our department apply stress psychological intervention methods to patients with ARF. Through analysis of the causes of psychological problems, health education, comfort communication, encouragement and support, and other measures, they can maximize patients' compliance and establish a healthy attitude.

### 4.1. Stress Psychological Intervention Can Improve Cardiopulmonary Function

For patients with ARF, ARF often leads to varying degrees of cardiac function and lung function damage, affecting the prognosis of patients. In this study, the experimental group had higher LVEF, FS, FEV_1_, FVC, and FEV_1_/FVC and lower LVMI. This shows that stress psychological intervention can significantly improve cardiopulmonary function. Stress psychological intervention follows the characteristics of ARF patients and converts signals into abstract concepts through the brain, which act on the endocrine system, nervous system, and immune system, so as to improve cardiopulmonary function. Stress psychological intervention uses simple and understandable language to introduce disease knowledge to ARF patients in detail, prompts patients to master the entire treatment and nursing process, and uses body language to comfort patients, so that patients can receive psychological support and comfort and gain the trust of patients, so as to improve the degree of treatment cooperation of patients. In addition, stress psychological intervention provides comprehensive interventions for ARF patients through the four aspects such as diagnosis, understanding, communication, and re-education. The nursing plan is more targeted, which increases the patient's enthusiasm for treatment and improves clinical symptoms. Clinically, we should communicate with ARF patients more, understand the basic situation of the patients, mobilize the enthusiasm for treatment, make them actively participate in their own management, and do a good job of nursing with enthusiasm and kindness, which plays an important role in speeding up the recovery of the disease.

### 4.2. Stress Psychological Intervention Can Reduce Negative Emotions

Anxiety and depression are the main parts of negative emotions, both of which are related to the occurrence and development of diseases. We found that after applying stress psychological intervention, the negative emotions of ARF patients were significantly reduced. Stress psychological intervention carries out a series of intervention plans based on the patients' own situation of ARF and based on the experience of our physicians for many years; we believe that when patients experience anxiety or depression, they should be encouraged to recall the happy things in life at this time and to listen to more relaxing music, so that patients can keep their body relaxed and happy; at the same time, the nursing staff can remind the patient to look at the natural scenery more, read more positive books, or see film and television works and encourage the patient to call the close family and friends; family members should be required to provide family support, and hence the importance of family care was emphasized to the patients' family members and they were urged to pay more attention to the psychological state of patients. These intervention plans are conducive for nurses to have a comprehensive understanding of the patient's psychological status, which can avoid the blindness of the traditional nursing model and is conducive to release anxiety, depression, and reduce the mental burden of patients, so as to establish the belief to overcome the disease and difficulties. In the process of stress psychological intervention, medical staff take the patients as the center and provide targeted care to the patients. The psychological counseling of ARF patients helps increase the communication between nurses and patients, understand the reasons for the formation of negative psychology, explain to them the harm of negative psychology, and take the initiative to ask and meet the needs of patients as much as possible, so as to encourage the patients to develop the habit of self-regulating emotions. At the same time, stress psychological intervention can alleviate various psychological stress responses in patients during treatment, adjust the patient's self-statement, encourage patients to establish a healthy state of mind, help them establish ideas that are conducive to recovery, and increase their confidence in recovery.

### 4.3. Stress Psychological Intervention Can Improve Self-Efficacy

Self-efficacy refers to the belief that people successfully implement and complete a certain behavior goal or face difficulties. It is a factor that determines human behavior and can significantly affect people's emotions and affect people's health outcomes. Generally speaking, the greater the self-efficacy an individual possesses, the greater the positive effect of persistence and effort on their behavior and the higher the level of mental health. More and more studies have shown that improving self-efficacy plays an important role in the management of chronic and mental illnesses [21]. Most patients with ARF are depressed and pessimistic, so psychological support is the key to alleviating their psychological pressure. In the process of stress psychological intervention, the care of family members and society can make ARF patients develop the courage to face life, increase the patients' sense of belonging to the society, and improve the patients' sense of self-efficacy. In this study, compared with conventional nursing intervention, stress psychological intervention has a more obvious effect on improving self-efficacy. This study uses various measures such as communication, health education, comfort and encouragement, and change of concepts to carry out stress psychological interventions on patients with ARF, conduct in-depth conversations according to different patients psychological state, and guide them to understand the importance of correct cognition and behavior, thus eliminating the influence of various unfavorable factors on patients and improving patients' sense of self-efficacy. In addition, medical staff conduct regular communication training for the family members of ARF patients, instructing family members to pay more attention to the patients' physical and mental condition and to provide psychological support to the patient, which can give full play to the patients' inherent potential, improve the patients' behavior, and enable the patients to develop the courage to face the disease and improve their sense of self-efficacy.

### 4.4. Stress Psychological Intervention Can Improve Quality of Life

After literature searches and clinical experience summary, nursing staff in our department applied stress psychological intervention to patients with ARF, and the results found that after the intervention, the living standard of patients was improved. This strategy takes patients as the center and implements comprehensive intervention in various aspects. By looking for the essential needs of patients with ARF, and focusing on the analysis and discussion of the causes of unreasonable problems, it is helpful for patients establish rational concepts and positive behavior patterns and establish confidence to overcome difficulties, enhance patients' self-management ability, and improve their living standards. In addition, stress psychological intervention can maximize nursing effectiveness as much as possible and has better intervention effects than conventional intervention methods. This method helps patients maintain a good state of mind by giving patients psychological intervention and increasing nurse-patient communication, and through reasonable music therapy and sports training, it can reduce the clinical symptoms of patients to a certain extent and improve the mental health and cognition of patients with ARF. There are significant improvements in thinking, treatment coordination, and living habits, thereby improving the quality of life of patients.

## 5. Conclusion

In summary, stress psychological intervention in patients with ARF can improve cardiopulmonary function, reduce negative emotions, improve self-efficacy, and improve quality of life. It is worthy of being widely used in clinical practice. The results of this study still need to be further verified by larger sample size data, and the long-term intervention effect needs to be discussed. We need to continue to collect more case information in the later stage to improve and supplement the study.

## Figures and Tables

**Figure 1:** Comparison of cardiac function between the two groups. Compared with the control group, ^*∗*^*P* < 0.05; compared with before intervention, #*P* < 0.05.

**Figure 2:** Comparison of lung function between the two groups. Compared with the control group, ^*∗*^*P* < 0.05; compared with before intervention, ^#^*P* < 0.05.

**Figure 3:** Comparison of negative emotions between the two groups. compared with the control group, ^*∗*^*P* < 0.05; compared with before intervention, #*P* < 0.05.

**Figure 4:** Comparison of self-efficacy between the two groups. Compared with the control group, ^*∗*^*P* < 0.05; compared with before intervention, ^#^*P* < 0.05.

**Figure 5:** Comparison of quality of life between the two groups. Compared with the control group, ^*∗*^*P* < 0.05; compared with before intervention, ^#^*P* < 0.05.

**Table 1:** Comparison of clinical data between the two groups (*n*, %).

Clinical data	Control group (*n* = 52)	Experimental group (*n* = 52)	*χ*^2^ value	*P* value
Age (years)				
<65	23 (44.23%)	25 (48.08%)	0.155	0.694
≥65	29 (55.77%)	27 (51.92%)		

Gender				
Male	28 (53.85%)	26 (50.00%)	0.154	0.695
Female	24 (46.15%)	26 (50.00%)		

Type				
Type I	32 (61.54%)	37 (71.15%)	1.077	0.299
Type II	20 (38.46%)	15 (28.85%)		

Cause of disease				
Chronic obstructive pulmonary emphysema	20 (38.46%)	21 (40.38%)	1.186	0.978
Severe or critical asthma	11 (21.15%)	9 (17.31%)		
Acute respiratory distress syndrome	7 (13.46%)	7 (13.46%)		
Sleep apnea syndrome	6 (11.54%)	8 (15.38%)		
Spontaneous pneumothorax	3 (5.77%)	4 (7.69%)		
Acute pulmonary infarction	3 (5.77%)	2 (3.85%)		
Other	2 (3.85%)	1 (1.92%)		

Level of education				
Junior high school and below	35 (67.31%)	32 (61.54%)	0.388	0.824
High school	13 (25.00%)	15 (28.85%)		
University and above	4 (7.69%)	5 (9.62%)		

## Data Availability

The data used and/or analyzed during the current study are available from the corresponding author.
